The article "A Multicriteria English Teaching Decision Model Based on Deep Learning" was published in 2022. Journal: Comput Intell Neurosci.

# A Multicriteria English Teaching Decision Model Based on Deep Learning

**DOI:** 10.1155/2022/9030626

**Published:** 2022-05-13

**Authors:** Jiachen Zhang

**Affiliations:** School of Foreign Languages, Fuzhou University of International Studies and Trade, Fuzhou 350202, China

## Abstract

In any stage of the teaching process, the teaching behavior depends on the decision of teachers. For English teachers, the English teaching decision level directly determines the course quality and the mining of learner potential. The existing studies only focus on a single teaching stage and involve one decision maker. The scientific level of decision is yet to be examined. Therefore, this paper develops a multicriteria English teaching decision (MCETD) model based on deep learning. Specifically, the author summarized the internalization and generation of MCETDs and expounded the generation mechanism of such decisions. Next, the problem of MCETD was described and mathematically modeled. After that, a neural network was constructed to weigh decision criteria and decision makers. In addition, the author explained how to comprehensively rank and generate MCETD schemes. Through experiments, the author obtained the information of decision matrix and preference ranking of decision schemes from decision makers and validated the effectiveness of the proposed model.

## 1. Introduction

In 2011, China released a new version of national English curriculum standard, calling English teachers to adjust their roles in the teaching process [1–5]. English teachers are urged to pursue the overall training goals of the course, after fully considering English application skills, English vocabulary and grammar, and English communication skills [6–9]. To ensure the sustainable development of English teaching, it is fundamental to arrange the English teaching tasks in each stage, integrate advantageous teaching resources, and enhance the effect of teacher-student interaction in class [10–13]. These measures can only be effectively implemented when teachers make a series of sound teaching decisions. In any stage of the teaching process, the teaching behavior depends on the decision of teachers [14, 15]. For English teachers, the English teaching decision level directly determines the course quality and the mining of learner potential. Thus, the only way to establish a classroom in line with practical teaching requirements is to continuously boost the awareness of English teachers for teaching decisions and optimize their teaching decision process.

Gao et al. [16] put forward a structural optimization approach for the intelligent decision support system based on the integration of the higher English teaching quality assessment model. Firstly, the structural optimization of the intelligent decision support system was discussed, after selecting different groups by the optimization strategy integrating the higher English teaching quality assessment model. Next, the structures of intelligent decision support systems with different features were optimized, using the higher English teaching quality assessment model. Finally, the experimental data on English teaching behavior were compared with the results of other classic optimization models.

The continuous development and application of artificial intelligence (AI) provides a new perspective for schools and teachers to reassess and configure physical education (PE) courses. Liu [17] explored the intelligence evaluation system for PE teaching based on the AI expert decision system. Firstly, the current situation of PE teaching evaluation systems was summarized, before presenting the definition and structure of the AI expert decision system; thence, index weighting was performed for the AI-based PE teaching evaluation system.

To avoid the uncertainties of technology, finance, and policy, Yong [18] suggested solving unconventional tasks, especially the development of language skills during foreign language learning, with an effective decision system [19]. João and Quadrado [20] demonstrated how decision analysis helps engineers better understand problems, highlighted the necessity of structured decision analysis, and advocated solving sustainability issues with multicriteria decision analysis. Yu and Li [21] proposed to aggregate dual hesitant fuzzy elements with several clustering operators, presented a multiobjective decision method under the dual fuzzy decision environment, and applied the method to assess teaching quality.

In summary, most researchers discussed the generation mechanism of objective decisions from the perspectives of the connotations, features, and influencing factors of multicriteria English teaching decision (MCETD). These discussions lay a profound theoretical foundation and provide new ideas for the research of MCETD generation mechanism.

Teaching decision ought to be a process involving multiple decision makers under multiple criteria. The existing studies only focus on a single teaching stage, failing to recognize teaching as a continuous and evolving process. The available measuring indices are too few to work in complex teaching scenarios. In addition, the teaching decisions that have been investigated are largely primary ones, involving only one decision maker. The scientific level of decision is yet to be examined.

Therefore, this paper develops an MCETD model based on deep learning. The weights were allocated and adjusted by learning and training the structure and samples of neural networks. In this way, the weights were determined more reasonably and reliably, resulting in correct decisions. The overall structure and detailed contents of this paper are as follows: (1) summing up the internalization and generation of MCETDs and expounding the generation mechanism of such decisions; (2) describing and mathematically modeling the MCETD problem; (3) proposing a neural network to weigh decision criteria and decision makers; and (4) providing a method to comprehensively rank and generate MCETD schemes. The proposed model was proved effective through experiments.

The research results enrich the theories and practical cases for further discussing the generation mechanism of teaching decisions and provide theoretical support and research ideas for the generation mechanism of English teaching decisions.

## 2. Problem Description and Mathematical Modeling

Based on scientific theories of English education and practice of English teaching, the current teaching decision can be optimized by mining the existing English teaching experience and verified through application in specific teaching scenarios. At present, the basic idea of English teaching is to convert teaching experience into teaching wisdom in four steps: the generation, application, reflection, and internalization of decisions. The teachers' understanding of decision generation and internalization depends on his/her teaching preferences. In general, decision internalization can be regarded as the acceptance of new teaching experience and the transformation of old teaching model to new teaching model. This paper divides the MCETD internalization and generation mechanism into four stages (Figure 1): generation stage, application stage, reflection stage, and internalization stage.

As shown in Figure 2, the premise of MCETD generation is that the decision makers must have the professional knowledge, teaching theories, and practical experience, which are necessary for preparing decision schemes. Besides, the decision makers must be able to analyze the teaching preferences, strengths, and weaknesses of the decision schemes of other decision makers. The final teaching decision scheme should not be discussed and generated by a single teacher under a single set of English teaching decision criteria. Otherwise, the final decision scheme would deviate from the actual teaching demand. Thus, the MCETD must actively discuss the interaction and sharing between every decision scheme and teachers, between teachers and students, and between functional departments of teaching at school.

For *m* known English teaching decision criteria, the criteria weight matrix can be expressed as *Q*=[*q*1, *q*2,…,*qm*]^*T*^(*m* > =2), where *q*_*j*_ is the weight of the *j*-th criteria. Let *q*^*l*^=[*q*^*l*^1, *q*^*l*^2,…,*q*^*l*^*m*]^*T*^ be the decision criteria weights of decision maker *r*^*l*^; $\mu ={\left[\mu 1,\mu 2,\ldots ,\mu t\right]}^{T}\left(t\underline{\geq }2\right)$ be the decision weight matrix of the *t*-th decision maker; *μ*_*l*_ be the decision weight corresponding to the *l*-th decision maker; *S*^*l*^=[*s*^*l*^1, *s*^*l*^2,…, *s*^*l*^*n*](*n* > =2) be the matrix of the overall preference ranking of the kl-th decision maker for mn English teaching decision schemes; *b*^*l*^1,…, *b*^*l*^*n* be the single point value of the ranking obtained through the normalization of *S*^*l*^, with *i*=1,…, *n*, *j*=1,…, *m*, and *l*=1,…, *t*; and *X*^*l*^=[*x*^*l*^*ij*]_*n*×*m*_ be the decision matrix given by decision maker *r*^*l*^, where *x*^*l*^*ij* is the score given by the l-th decision maker for decision scheme *E*_*i*_ under criterion *D*_*j*_, *i*=1,…, *n*, *j*=1,…, *m*, and *l*=1,…, *t*.

For complex MCETD problems, this paper firstly transforms the decision criteria scores in different forms, i.e., the decision matrix *X*^*l*^=[*x*^*l*^*ij*]_*n*×*m*_ into comparable utilities, i.e., a decision matrix *Y*^*l*^=[*Y*^*l*^*ij*]_*n*×*m*_ of single point values in the range of [0, 1]. By the simple weighted sum method, the distance from the composite scores given by each decision maker for decision schemes to the preference ranking *b*^*l*^*i* can be calculated by

(1) $$\begin{array}{c} DIS_{i}^{l}={\left(\sum_{j=1}^{m}q_{j}^{l}y_{ij}^{l}-b_{i}^{l}\right)}^{2},i=1,\ldots ,n,l=1,\ldots ,t. \end{array}$$

To minimize *DIS*_*i*_^*l*^, it is necessary to optimize the decision model in search of the ideal criteria weights. The decision model can be established as

(2) $$\begin{array}{c} \min={\left(\sum_{j=1}^{m}q_{j}^{l}y_{ij}^{l}-b_{i}^{l}\right)}^{2},i=1,\ldots ,n,l=1,\ldots ,t,\\ s.t\\ \sum_{j=1}^{m}q_{j}^{l}=1\\ 0\leq q_{j}^{l}\leq 1,j=1,2,\ldots ,m. \end{array}$$

Solving formula (2), the distance matrix between composite scores *E*_1_, *E*_2_,…, *E*_*n*_ and preference ranking *b*^*l*^*i* can be given as

(3) $$\begin{array}{c} dis=\left(\begin{array}{ccc} dis_{1}^{1} & \cdots & dis_{1}^{t}\\ \vdots & \ddots & \vdots \\ dis_{n}^{1} & \cdots & dis_{n}^{t} \end{array}\right). \end{array}$$

During the MCETD process, the weight of each decision maker depends on his/her importance. For each given decision scheme, it is necessary to minimize the *DIS* of all decision makers, with the optimal value being zero. If the optimization objective of the decision model is set to zero for actual teaching, the teaching effect would be suboptimal, and even negative. Hence, the objective was set to 10^−4^. Then, a mathematical model can be established based on decision weights:

(4) $$\begin{array}{c} min{\left(l=1\sum^{t}\mu_{l}^{*}DIS^{l}-10^{-4}\right)}^{2},\mu_{l}^{*}>0,l=1,\ldots t. \end{array}$$

Based on formula (4), the weight *μl*^*∗*^ is solved. In the MCETD, decision weights should satisfy

(5) $$\begin{array}{c} \sum_{l=1}^{t}\mu_{l}=1,\\ 0\leq \mu_{l}\leq 1,l=1,\ldots t. \end{array}$$

Normalizing the obtained weights, the final decision weights can be obtained as

(6) $$\begin{array}{c} \mu_{l}=\frac{{\bar{\mu }}_{l}}{\sum_{l=1}^{t}{\bar{\mu }}_{l}},l=1,\ldots t. \end{array}$$

As stated above, the composite scores of English teaching decision schemes were processed by the weighted sum method, which mainly discloses the linear relationship between the teaching decision matrix and criteria weights. The preference ranking of decision schemes given by decision makers can be viewed as the desired result of decision makers. Hence, the smaller the *DIS*, the better the decisions. The criteria weights at the minimum *DIS* are the criteria weights of the MCETD.

To sum up, the linear adaptive neural network was adopted, with the attributes of decision schemes as inputs and composite score as the output. Using the function of the neural network for memorizing decision preference ranking, positive network weights were trained and normalized as the attribute weights of multiattribute decision making. For expert weights, the distance variable *DIS* was imported to the network, and the output was expected to be 0.0001. Similarly, positive network weights were trained and normalized as the expert weights for group decision making.

## 3. Deep Learning-Based Weighting

### 3.1. Solving Criteria Weights

The English teaching decision model formulas (2) and (3) aim to minimize *DIS*. This is similar to the least mean square error (LMSE) algorithm in deep learning. The goal is to keep the actual output of the proposed neural network consistent with the desired output, as much as possible. In this section, the composite scores given by each decision maker to English teaching decision schemes are taken as the actual output of the neural network, and the preference ranking is taken as the desired output. The difference between the actual and desired output was defined as the training objective of the neural network. The ideal neural network was obtained by adjusting the network weights and iterative training. Here, the weights are trained by an adaptive linear neural network, where each node is a linear function.

Figure 3 presents the structure of the proposed linear neural network. It can be seen that the proposed linear neural network consists of an input layer of *m* nodes and an output layer of 1 node. Let *n* be the number of English teaching decision samples. Without considering network thresholds, the output of the output layer under the samples can be expressed as

(7) $$\begin{array}{c} OI_{i}^{l}=\sum_{j=`1}^{m}y_{ij}^{l}q_{j}^{l},i=1,2,\ldots ,n,l=1,\ldots ,t. \end{array}$$

Let *u*(.) be the activation function. The output *OO*^*l*^*i* of the output layer can be calculated by

(8) $$\begin{array}{c} OO_{i}^{l}=u\left(OI_{i}^{l}\right),i=1,2,\ldots ,n,l=1,\ldots ,t. \end{array}$$

The proposed network adopts the following linear function:

(9) $$\begin{array}{c} OO_{i}^{l}=u\left(OI_{i}^{l}\right)=\sum_{j=`1}^{m}y_{ij}^{l}q_{j}^{l},i=1,2,\ldots ,n,l=1,\ldots ,t. \end{array}$$

Let *b*^*l*^*i* be the desired output of the network. Then, the quadratic error function of the network for sample *i* can be expressed as

(10) $$\begin{array}{c} {\text{ERROR}}_{i}^{l}=\frac{1}{2}\left(b_{i}^{l}-OO_{i}^{l}\right)=\frac{1}{2}r_{i}^{2},i=1,2,\ldots ,n,l=1,\ldots ,t. \end{array}$$

For *n* training samples, the total error can be calculated by

(11) $$\begin{array}{c} {\text{ERROR}}^{l}=\sum_{i=1}^{n}{\text{ERROR}}_{i}^{l}=\frac{1}{2}\sum_{i=1}^{n}{\left(b_{i}^{l}-OO_{i}^{l}\right)}^{2}=\frac{1}{2}\sum_{i=1}^{n}r_{i}^{2},i=1,2,\ldots ,n,l=1,\ldots ,t. \end{array}$$

The *ERROR* can be ensured by adjusting network weights:

(12) $$\begin{array}{c} \min\;{\text{ERROR}}^{l}=\sum_{i=1}^{n}{\text{ERROR}}_{i}^{l}=\frac{1}{2}\sum_{i=1}^{n}{\left(b_{i}^{l}-OO_{i}^{l}\right)}^{2}=\frac{1}{2}\sum_{i=1}^{n}r_{i}^{2},i=1,\ldots ,n,l=1,\ldots ,t. \end{array}$$

Following the Widrow–Hoff learning rule, this paper corrects the weighted coefficients of the proposed network. The LMSE algorithm mainly adopts the fastest gradient descent to make network weights change in the negative gradient direction of *ERROR*. The weighting coefficients of network nodes can be modified by

(13) $$\begin{array}{c} \Delta q_{j}^{l}=-\delta \frac{\partial {\text{ERROR}}_{i}^{l}}{\partial q_{j}^{l}},i=1,\ldots ,n,j=1,\ldots ,m,l=1,\ldots ,t,\\ \frac{\partial {\text{ERROR}}_{i}^{l}}{\partial q_{j}^{l}}=\frac{\partial {\text{ERROR}}_{i}^{l}}{\partial OO_{i}^{l}}\frac{\partial OO_{i}^{l}}{\partial OI_{i}^{l}}\frac{\partial OI_{i}^{l}}{\partial q_{j}^{l}}\\ =-\left(b_{i}^{l}-OO_{i}^{l}\right)y_{ij}^{l},i=1,\ldots ,n,j=1,\ldots ,m,l=1,\ldots ,t\\ =-r_{i}^{l}y_{ij}^{l}. \end{array}$$

Thus,

(14) $$\begin{array}{c} \Delta q_{j}^{l}=\delta r_{i}^{l}y_{ij}^{l},i=1,\ldots ,n,j=1,\ldots ,m,l=1,\ldots ,t. \end{array}$$

The proposed network learning algorithm can be implemented in the following steps.

**Step 1 .**

Initialize neural network parameters and set the initial weights *q*^*l*^=[1/*m* … 1/*m*]_1×*m*^*T*^_.

**Step 2 .**

Input the English teaching decision samples and desired output, i.e., the composite scores of decision schemes and preference ranking. To ensure that the network weights corrected during network training are all positive, the desired output can be adjusted as

(15) $$\begin{array}{c} \psi_{i}^{l}=b_{i}^{l}+\text{min}\frac{1}{m}\sum_{j=1}^{m}y_{ij}^{l},i=1,\ldots ,n,l=1,\ldots ,t. \end{array}$$

According to the preference ranking of MCETDs, the final result will not be affected if the desired output of each sample is adjusted and superposed with a constant.

**Step 3 .**

Compute the actual output of the output layer.

**Step 4 .**

Compute network error. If the LMSE of the output satisfies the error precision required for network output, then

(16) $$\begin{array}{c} \max\left|OO_{i}\left(p\right)-OO_{i}\left(p+1\right)\right|\leq \sigma ,i=1,\ldots ,n. \end{array}$$

If the error precision is satisfied and the trained weights are integers, then terminate the iterative training of the network; otherwise, go to Step 5.

**Step 5 .**

Adjust the weight coefficient *q*^*l*^*j*(*p*) between the input layer and the output layer.

**Step 6 .**

Return to Step 3. Terminate the iterative training of the network when the maximum number of training is reached and the trained weights are greater than zero.

**Step 7 .**

Normalize the network weights obtained through the final training, i.e., obtain the criteria weights of English teaching decisions *q*^*l*^=[*q*^*l*^1, *q*^*l*^2, ..., *q*^*l*^*m*]^*T*^.

Figure 4 shows the execution flow of the neural network algorithm.

### 3.2. Solving Weights of Decision Makers

At present, the environment and model of English teaching are increasingly complex, and the English learning resources are quickly expanding. As a result, many English teaching decision problems become more and more complicated. Different decision makers are of different levels of importance in English teaching decision process, owing to their disparity in learning background, professional level, and personal preferences. Hence, the decisions of different decision makers take up different proportions in the final decision scheme. Therefore, it is of great practical significance to determine the level of importance of each decision maker in MCETD, i.e., the weight of each decision maker.

To fulfil the above task, this paper solves the weight of each decision maker by the proposed neural network and assigns a precise weight to each decisions scheme. When solving the decision criteria weights, each decision maker looks for the optimal solutions to multiple decision schemes. Hence, solving the weights of decision makers is a multiperson, single-objective process. In the end, all schemes need to be combined to obtain the optimal solution.

Based on the neural network training in the preceding section, the criteria weights given by each decision maker for decision schemes can be obtained after completing the training of *t* decision makers:

(17) $$\begin{array}{c} q=\left(\begin{array}{ccc} q_{1}^{1} & \cdots & q_{m}^{1}\\ \vdots & \ddots & \vdots \\ q_{1}^{l} & \cdots & q_{m}^{l} \end{array}\right),l=1,\ldots ,t. \end{array}$$

For the decision criteria weights of a single decision maker, the desired output of samples is defined as the decision maker's preference ranking of each scheme. Since DIS is taken as the network input to determine the weights of decision makers, the desired output of the network is the optimal solution to be obtained for the actual teaching situation. The training process of the proposed network is consistent with that of the criteria weights. The obtained trained network weight matrix can be expressed as *μ*^*∗*^=[*μ*1^*∗*^, *μ*2^*∗*^,…*μl*^*∗*^,…*μt*^*∗*^]^*T*^. Considering the actual teaching situation, the desired output is set to 10^−4^ to ensure the existence of weights. The final decision weight can be expressed as

(18) $$\begin{array}{c} \mu_{l}=\frac{\mu_{l}^{*}}{\sum_{l=1}^{t}\mu_{l}^{*}},l=1,\ldots ,t. \end{array}$$

After obtaining the decision weights and the criteria weights corresponding to each decision maker, it is necessary to solve the composite criteria weight by

(19) $$\begin{array}{c} q_{j}=\sum_{l=1}^{t}\mu_{l}q_{j}^{l},l=1,\ldots ,t. \end{array}$$

### 3.3. Composite Ranking of Decision Schemes

When the planned decision matrix *Y*^*l*^=[*y*^*l*^*ij*]_*n*×*m*_ of single point values is known, the composite score *ZH*=[*ξ*1,…*ξi*,…,*ξn*]^*T*^ can be obtained through simple weighting:

(20) $$\begin{array}{c} \zeta_{i}=\sum_{l=1}^{t}\sum_{j=1}^{m}y_{ij}^{l}\mu_{l}q_{j},i=1,\ldots ,n,j=1,\ldots ,m,l=1,\ldots ,t. \end{array}$$

The final composite ranking of English teaching decisions is obtained by sorting the schemes in descending order of *ζi*.

## 4. Experiments and Result Analysis

Five alternative English teaching decision schemes *E*_1_, *E*_2_, *E*_3_, *E*_4_, and *E*_5_ were provided, each of which contains four decision criteria indices *DC*_1_, *DC*_2_, *DC*_3_, and *DC*_4_. Suppose all four decision criteria are based on the teaching effect. The score of each criterion depends on multiple teaching preferences and teaching forms. Three experts *r*^1^, *r*^2^, and *r*^3^ were invited to make decisions about the five English teaching decisions. Decision criterion *DC*_1_ evaluates each decision scheme by preference ranking; decision criterion *DC*_2_ evaluates each decision scheme by teaching plan; decision criterion *DC*_3_ evaluates each scheme by teaching interaction; and decision criterion *DC*_34_ evaluates each scheme by teaching effect.  Table 1 lists the information of the decision information for each scheme.

It can be seen that the preference ranking of expert *r*^1^ for the English teaching decision schemes was 2-1-3-5-4, and the normalized preference matrix was [0.75 1 0.5 0 0.25]^T^. The preference ranking of expert *r*^2^ for the English teaching decision schemes was 3-5-2-1-4, and the normalized preference matrix was [0.5 0 0.75 1 0.25]^T^. The preference ranking of expert *r*^3^ for the English teaching decision schemes was 1-3-4-2-5, and the normalized preference matrix was [1 0.5 0.25 0 0.25 0]^T^.  Table 2 shows the results of network learning.

To verify the effectiveness of our neural network in English teaching decision, the network structure was initialized and trained 25 times by the Trainrp function. The mean squared error (MSE) of the network reached the preset error requirement, and the trained network converged. In this case, the MSE reached 8.2517e–05.  Figure 5 shows the training convergence of the neural network.  Figure 6 shows the linear regression results of our network.

When the network training approached convergence, the error between the actual output and desired output peaked at 0.0154 and minimized at 0.0002. When the network testing approached convergence, that error peaked at 0.0411 and minimized at 0.0005. Compared with the results of the other networks, the training error of our network was close to the test error. Hence, the proposed adaptive linear neural network performs well and provides a simple, effective, and feasible way to evaluate English teaching decisions.

The above analysis reveals that after the neural network is applied to the MCETD process, the self-learning function of the neural network manages to adjust weights automatically. With the continuous growth of learning rounds and sample size, a law is formed in terms of weight update, and the learning model can be determined for the network. Facing the increasing data on MCETD schemes, the trained network can be applied directly to learn the data and rank the MCETD schemes comprehensively. The weights allocated by the neural network are objective and accurate. Our neural network makes it easier to complete the MCETD amidst numerous schemes.

## 5. Conclusions

This paper explores the MCETD model based on deep learning. After summing up the internalization and generation of MCETDs, the author explained the generation principle of MCETDs, described the MCETD problem, and provided the corresponding mathematical model. Then, a neural network was established to compute the weights of decision criteria and decision makers. After that, an approach was presented for composite ranking of MCETD schemes. Through experiments, the author obtained the information of decision matrix and preference ranking of decision schemes from decision makers and summarized the learning results, convergence, and linear regression results of the proposed neural network. The closeness between the training error and testing error suggests that the proposed network is a simple, effective, and feasible tool to evaluate English teaching decisions.

Admittedly, there are several defects with this research. For example, the methodology is mainly qualitative, lacking data support. Besides, the limited sample size should be expanded in the follow-up research. The proposed mechanism for internalizing, externalizing, and sharing MCETD is not only a generation mechanism of teaching decisions but also an exploratory tool for teaching decision generation. Further research is needed to devise a universal generation mechanism for teaching decisions.

## Figures and Tables

**Figure 1:** Internalization and generation of MCETDs.

**Figure 2:** Generation principle of MCETDs.

**Figure 3:** Structure of the proposed linear neural network.

**Figure 4:** Flow of neural network algorithm.

**Figure 5:** Convergence of neural network training.

**Figure 6:** Linear regression results.

**Table 1:** Information of decision matrix and preference ranking of decision schemes.

Scheme		*E*_1_	*E*_2_	*E*_3_	*E*_4_	*E*_5_
*r* ^1^	*DC*_1_	2	6	3	5	2
	*DC*_2_	[3.2, 4.5]	[3.5, 4.2]	[3.1, 3.7]	[2.5, 3.9]	[3.3, 4.2]
	*DC*_3_	Good	Very good	Good	Poor	Very good
	*DC*_4_	[*t*_2_, *t*_4_]	[*t*_3_, *t*_6_]	[*t*_1_, *t*_5_]	[*t*_2_, *t*_6_]	[*t*_2_, *t*_7_]
	Ranking	2	1	3	5	4

*r* ^2^	*DC*_1_	6	3	2	5	1
	*DC*_2_	[2.5, 3.3]	[3.7, 4.3]	[3.6, 3.9]	[3.2, 3.8]	[4.3, 4.7]
	*DC*_3_	Very good	Good	Poor	Very good	Good
	*DC*_4_	[*t*_2_, *t*_7_]	[*t*_1_, *t*_4_]	[*t*_3_, *t*_6_]	[*t*_2_, *t*_8_]	[*t*_4_, *t*_6_]
	Ranking	3	5	2	1	4

*r* ^3^	*DC*_1_	5	3	6	4	2
	*DC*_2_	[2.5, 3.1]	[2.9, 3.7]	[4.3, 4.8]	[3.5, 4.2]	[2.8, 4.6]
	*DC*_3_	Poor	Very good	Good	Good	Poor
	*DC*_4_	[*t*_2_, *t*_5_]	[*t*_4_, *t*_8_]	[*t*_1_, *t*_3_]	[*t*_4_, *t*_6_]	[*t*_5_, *t*_7_]
	Ranking	1	3	4	2	5

**Table 2:** Results of network learning.

Sample number	1	2	3	4	5	6
Desired output	0.4305	0.3627	0.4015	0.4268	0.3924	0.2859
Actual output	0.4927	0.3624	0.3906	0.4315	0.4471	0.4827
Relative error	0.0026	0.0007	0.0081	0.0074	0.0062	0.0092

Sample number	7	8	9	10	11	12

Desired output	0.4172	0.3952	0.7485	0.3928	0.3714	0.5629
Actual output	0.4638	0.3315	0.4052	0.6829	0.6642	0.5837
Relative error	0.0017	0.0082	0.0006	0.0047	0.0036	0.0095

## Data Availability

The data used to support the findings of this study are available from the corresponding author upon request.
